# Electroacupuncture and Moxibustion Modulate the BDNF and TrkB Expression in the Colon and Dorsal Root Ganglia of IBS Rats with Visceral Hypersensitivity

**DOI:** 10.1155/2021/8137244

**Published:** 2021-09-28

**Authors:** Duiyin Jin, Yanan Liu, Siyi Lv, Qin Qi, Mei Li, Yuanyuan Wang, Xiaomei Wang, Huangan Wu

**Affiliations:** ^1^Yueyang Clinical Medical College, Shanghai University of Traditional Chinese Medicine, Shanghai 200437, China; ^2^Shanghai Research Institute of Acupuncture and Meridian, Shanghai University of Traditional Chinese Medicine, Shanghai 200030, China; ^3^Key Laboratory of Acupuncture and Immunological Effects, Shanghai University of Traditional Chinese Medicine, Shanghai 200030, China

## Abstract

**Objective:**

To evaluate the effects of electroacupuncture and moxibustion on brain-derived neurotrophic factor (BDNF) and its receptor tyrosine kinase receptor B (TrkB) protein and mRNA expressions in the colon and dorsal root ganglia of IBS rats with visceral hypersensitivity and to explore their underlying therapeutic mechanisms.

**Method:**

Forty Sprague Dawley rats were randomly divided into normal, model, model + mild moxibustion (MM), model + electroacupuncture (EA), and model + pinaverium bromide (PB) groups, with eight rats in each group. Chronic visceral hypersensitive IBS rat models were established by colorectal distension (CRD) with mustard oil clyster. Rats in the MM and EA groups, respectively, received moxibustion and electroacupuncture treatments on the Tianshu (ST25) and Shangjuxu (ST37) acupoints once daily for 7 days, and rats in the PB group received pinaverium bromide by oral gavage once daily for 7 consecutive days. After treatment, rats underwent abdominal withdrawal reflex (AWR) scoring under CRD and colon histopathological examination. Immunohistochemistry and real-time quantitative PCR (RT-qPCR) were used to study the protein and mRNA expressions of BDNF and TrkB in the rat colon and dorsal root ganglia.

**Results:**

Compared with the normal group, AWR scores and body weight were clearly increased in the model group rats (both *P* < 0.01). The body weights were significantly elevated (*P* < 0.01, *P* < 0.05), but the AWR scores were reduced (*P* < 0.05, *P* < 0.01), after electroacupuncture and mild moxibustion treatment. Compared with levels in normal rats, BDNF and TrkB protein and mRNA expressions were significantly elevated in the IBS model rats (*P* < 0.01) but were downregulated after mild moxibustion, electroacupuncture, and Western medicine treatment (*P* < 0.01).

**Conclusion:**

Electroacupuncture and moxibustion improved visceral hypersensitivity of IBS rats possibly by reducing BDNF and TrkB protein and mRNA expressions in the colon and dorsal root ganglia.

## 1. Introduction

Irritable bowel syndrome (IBS) is a chronic functional gastrointestinal disorder with a syndrome of persistent or recurrent episodes of intestinal disorder. It is characterized by abdominal pain, abdominal distension, altered bowel habits, and/or character of stool that severely affect the quality of patients' life. At present, the pathogenesis of IBS has not yet been fully elucidated. Most studies suggest that IBS is related to the interaction of various factors including genes, diet, psychosocial factors, mucosal immunity and inflammation, intestinal flora disorders, gastrointestinal motility abnormalities, and brain-gut axis dysfunction, causing visceral hypersensitivity and manifesting as the corresponding symptoms [1–3].

Brain-derived neurotrophic factor (BDNF) is a neurotrophic protein widely distributed in the nervous system and is involved in neuronal differentiation, development, and repair and has the effect of causing pain and sensitivity in the nervous system [4, 5]. After being synthesized in primary sensory neurons, BDNF is transported to the primary afferent nerve terminals of the spinal cord dorsal horn, where it is involved in the regulation of pain hypersensitivity caused by different pain stimuli [6]. BDNF does not only present in the nervous system but also expresses in peripheral tissues, such as the intestine and pancreas [7, 8], and especially in the intestinal epithelium, myenteric plexus, and submucosal plexus of the colon. The fecal supernatants (FSN) from diarrhea-predominant IBS patients significantly increase BDNF mRNA and protein levels in colonic epithelial cells of humans and mice [9]. BDNF interacts with substance P (SP), nerve growth factor, and calcitonin gene-related peptide (CGRP) to regulate intestinal sensation and affect colon sensitivity [10]. Studies found that moderate amounts of BDNF can maintain the normal function of sensory nerves; however, abnormal elevation of BDNF can lead to a variety of pain-related sensations, such as chronic pain, inflammatory pain, and visceral pain [11].

A study has found that BDNF plays an important role in IBS pathogenesis and visceral sensitivity through binding with its high-affinity receptor of tyrosine receptor kinase B (TrkB) [12]. Currently, no effective Western medicine methods are available for IBS treatment. Although drugs such as pinaverium bromide and probiotics can relieve the symptoms, the long-term maintenance effect is unsatisfactory. Acupuncture and moxibustion are important parts of traditional Chinese medicine to alleviate visceral hypersensitivity and have good effects on improving the clinical symptoms of IBS patients, such as abdominal pain and bloating, as well as improving their quality of life [13–15]. However, the therapeutic mechanisms of acupuncture and moxibustion remain unclear. This study aimed to detect the expression of BDNF and TrkB in the colon and spinal cord of IBS rats and evaluate the regulatory effects and therapeutic mechanisms of acupuncture and moxibustion for visceral hypersensitivity in IBS.

## 2. Materials and Methods

### 2.1. Experimental Animals

40 neonatal male Sprague Dawley (SD) rats aged five days of clean grade were provided by the Laboratory Animal Center of the Shanghai University of Traditional Chinese Medicine (Shanghai, China). Each litter of neonatal rats and a female lactating rat that had free access to water and food were housed in a cage. The animal housing environment provided a 12-hour light/dark cycle at 20 ± 2°C room temperature and 50–70% indoor humidity. After adaptive feeding, experiments were conducted in neonatal SD rats 8 days after birth. All experiment procedures were performed in strict accordance with the guidelines provided by the National Institutes of Health for the Care and Use of Laboratory Animals, and the animal protocol was approved by the Animal Care and Use Committee of the Shanghai University of Traditional Chinese Medicine.

### 2.2. IBS Modeling and Identification

Colorectal distension (CRD) and intracolonic injection of mustard oil were used to establish the rat model of visceral hypersensitivity in IBS [16]. In this study, a hand-made saccule coated with a small amount of vaseline was slowly inserted from anus to the descending colon along the colorectal physiological curvature for approximately 2 cm. Saccule distension was made by inflating with 0.5 mL air for 1 minute followed by deflation. The same stimulation was repeated once after 30 min. The above procedures were conducted once a day for 14 consecutive days. Then, the rats continued feeding until postnatal week 6 and were intracolonically injected with 0.2 mL of 4% mustard oil daily for 14 consecutive days, with an injection depth of approximately 6–8 cm. Subsequently, abdominal withdrawal reflex (AWR) scoring under CRD was performed to evaluate their sensitivity to CRD stimulation to confirm successful modeling.

### 2.3. Abdominal Withdrawal Reflex (AWR) Scoring

AWR scoring was conducted by the method of Al-Chaer et al. [16] to evaluate behavioral changes in rats before and after treatment. All rats were fasted with free access to water for 8–12 hours before the AWR scoring. The balloon was connected to a desktop sphygmomanometer and syringe through a three-way valve to provide distension with constant pressure. The balloon was slowly inserted into the rectum from the anus and reached the descending colon of the rat. This was followed by inducing pain by colorectal distension at 20, 40, 60, and 80 mmHg. Each CRD scoring lasted approximately 20 seconds every 3 minutes, and each rat was evaluated 3 times to obtain the mean value as the final score for analysis. AWR scoring criteria were as follows: score 0, no behavioral response to CRD; score 1, brief head movement followed by immobility during CRD; score 2, mild contraction of the abdominal muscles but no lifting; score 3, strong contraction of the abdominal muscles and lifting of the abdomen without lifting of the pelvic structure and scrotum; and score 4, body was arched and lifting of the pelvis and scrotum [16].

### 2.4. Animal Grouping and Treatment

Laboratory animal treatments are in accordance with the International Association for the Study of Pain (IASP) guidelines. All 8-day-old neonatal rats were randomly divided into the normal group (*n* = 8) and IBS modeling group (*n* = 32). Rats in the normal group were routinely fed and housed without any stimulation; rats in the IBS modeling group were given CRD stimulation and intracolonically injected with mustard oil as described above. After the model was successfully established, 32 rats in the IBS modeling group were randomly divided into model group, mode + mild moxibustion (MM) group, model + electroacupuncture (EA) group, and model + pinaverium bromide (PB) group, 8 rats in each group.

In the MM group, rats were received moxibustion treatment on bilateral Tianshu (ST25) and Shangjuxu (ST37) acupoints [17]; special moxa sticks (Nanyang Hanyi Moxa Co., Ltd., Nanyang, Henan province, China) with a diameter of 0.5 cm were ignited and suspended at approximately 2–3 cm above the acupoints simultaneously for 10 minutes [18–20], once daily for 7 consecutive days. In the EA group, a disposable sterile acupuncture needle (0.25 mm × 25 mm; Suzhou Medical Appliance Factory, Jiangsu Province, China) was used for acupuncture at a depth of 5 mm on bilateral ST25 and ST37 acupoints and was connected to HANS-100A EA device (Nanjing Jisheng Medical Treatment Technology Co., Ltd., Jiangsu Province, China), with dilatational wave, 2/10 Hz frequency, and 1 mA intensity, 20 minutes for each time [19, 20], once daily for 7 consecutive days. Rats in the PB group received pinaverium bromide solution (State Food and Drug Administration, China, Approval number: H20120127) following the 1 : 0.018 of adult human (70 kg body weight)-to-rat (200 g body weight) ratio [21] by gavage daily for 7 consecutive days.

### 2.5. Sample Collection

After AWR scoring, all rats were weighed and anesthetized by intraperitoneal injection with 2% pentobarbital sodium (0.2 mL/100 g) and were then fixed on the dissection bench to open the abdominal cavity. Approximately 6–8 cm of colon tissue was collected 2 cm above the anus. The colon sample was cut longitudinally and rinsed with normal saline followed by fixing part of the colon sample in 4% paraformaldehyde solution and preserving the remaining sample at −80°C in a freezer for later experiments. Then, rats were sacrificed by cervical dislocation to reduce pain, and the spinal dorsal root ganglia at L6–S2 [17, 20, 22] were rapidly removed and preserved at −80°C in a freezer for later detection.

### 2.6. General Conditions in Rats

Mental state, fur appearance, dietary change, defecation, body weight, responsiveness, and activity of rats were monitored.

After IBS modeling was accomplished, AWR scoring was compared before and after each treatment to observe any behavioral changes in different groups of rats.

### 2.7. Histological Analysis

The colon tissues fixed in 4% paraformaldehyde solution were dehydrated, paraffin-embedded, and sectioned at a 4 *μ*m thickness. The sections were deparaffinized in xylene I and II solutions for 15 min each and rehydrated from 100%, 95%, 90%, 80%, and 70% ethanol (5 min each) in double-distilled water (5 min each for 2 times on a shaker) followed by staining in hematoxylin solution for 3 min and rinsing in running water for 10 min. After differentiating in 1% hydrochloric acid alcohol for 3 s and bluing in running water for 10 min, the tissue section was stained in eosin solution for 2 min followed by dehydrating from 70%, 80%, 90%, 95% (2 min each) to 100% ethanol for 5 min each, clearing in xylene I and II solutions for 15 min each, and mounting coverslips on the glass slides using appropriate amounts of neutral gum. After drying, the histopathological changes of colon tissues in different group rats were observed under a light microscope (BH2; Olympus, Tokyo, Japan).

### 2.8. Immunohistochemistry to Detect BDNF and TrkB Protein Expression

The paraffin sections of colon and dorsal root ganglia tissue were deparaffinized in xylene I and II solutions for 10 min each and rehydration in 100%, 95%, 85%, and 75% ethanol for 5 min. After washing with PBS 5 min each for 2 times on a shaker, tissue sections were immersed in 0.01 M citrate buffer (pH 6.0) and heated in a microwave at 98°C for 2.5 min, 1.5 min, and 1 min, with 15-min intervals for antigen retrieval. After cooling down to room temperature, tissue sections were placed in 1% H_2_O_2_ for 10 min, washed 3 times in PBS for 3 min each, and blocked in 5% bovine serum albumin at 37°C for 20 min. The tissue sections were individually incubated with 20 *μ*L primary antibodies (1 : 200 anti-BDNF antibodies, 1 : 25 anti-TrkB antibodies; Abcam, USA) overnight at 4°C. Next day, after 3 washes in PBS for 3 min each, the tissue sections were incubated with 20 *μ*L biotin-labeled secondary antibody (goat anti-rabbit IgG, 1 : 100; Wuhan Boster Bio-Engineering Co., Ltd., Wuhan, China) at 37°C for 30 min followed by washing in PBS 3 times for 3 min each. After incubation with biotin-labeled avidin solution at 37°C for 30 min, the sections were washed with PBS 3 times for 3 min each and subsequently incubated with DAB for color development. The sections were rinsed in running water for 10 min, counterstained with hematoxylin solution for 30 s, rinsed in running water again, blued in hydrochloric acid alcohol for 2 s, followed by washing in water, and were dehydrated, cleared, and mounted with neutral gum. Immunohistochemistry of colon tissue was observed under a light microscope (BH2; Olympus, Tokyo, Japan).

### 2.9. RT-qPCR to Detect BDNF and TrkB mRNA Expression

Total RNAs were extracted from colon and dorsal root ganglia tissues using TRIzol reagent (Invitrogen) followed by pipetting 2 *μ*L extracted RNA into a 1.5 mL centrifuge tube containing 8 *μ*L DEPC water, 0.5 *μ*L RNase inhibitor (50 U/*μ*L), and 2 *μL* (50 pM/*μ*L) random primers for reverse transcription and cDNA synthesis at 65°C in a water bath for 5 min. After standing at room temperature for 10 min, the mixtures were centrifuged at 5,000*g* for 5 s, then adding 0.5 *μ*L RNase inhibitor (50 U/*μ*L), 4 *μ*L 5 × buffer (Invitrogen), 2 *μ*L dNTP Mix (10 mM/each), and 1 *μ*L reverse transcriptase (AMV) (200 U/*μ*L) to the above reaction system to achieve a final reaction volume of 12.5 *μ*L. The samples were allowed to reaction for 1 h at 40°C in a water bath followed by 90°C for 5–10 min, ice bath for 5 min, and high-speed centrifuging at 5,000*g* for 5 s before PCR amplification. The RT-qPCR reaction system contained 5 *μ*L water, 8 *μ*L 2 × SYBRGREEN PCR mix, 1 *μ*L forward primer (10 pM/*μ*L), 1 *μ*L reverse primer (10 pM/*μ*L), and 1 *μ*L cDNA template. The RT-qPCR conditions were 95°C denaturation for 2 min, 40 cycles of 94°C denaturation for 10 s, 60°C annealing for 10 s, and 72°C elongation for 40 s. RT-qPCR was performed in a 7300 Real-Time PCR System (Applied Biosystems) to analyze the optical densities of the stripes, which were corrected by GAPDH to obtain the relative optical densities of the target genes.

### 2.10. Statistical Analysis

SPSS 20.0 software (IBM SPSS Inc., Chicago, IL, USA) was used for data statistics and analysis. The normally distributed data were presented as mean ± standard deviation ($\bar{x}\pm s$), and one-way ANOVA was used for comparison among groups. The least significant difference (LSD) method was used for multiple comparisons if the variances were homogeneous, and Dunnett's T3 method was performed if the variances were not homogeneous. Non-normally distributed data were presented as median (minimum, maximum), and the nonparametric Kruskal–Wallis test was used for the comparison between groups. The test standard was *α* = 0.05. *P* < 0.05 was considered a statistically significant difference.

## 3. Results

### 3.1. General Conditions of Rats in Each Group

Rats in the normal group were normal in food uptake and active and had white and well-groomed fur, stool with appropriate hardness, and clean perianal skin and fur. Rats in the model group were irritable and had poor appetite, reduced food uptake, slow movement, dry and sparse fur, watery stool, and dirty perianal skin. Rats in the MM, EA, and PB groups had different degrees of improvement in food uptake, grooming, responsiveness, and mobility, with most of the formed feces and occasionally contaminated perianal skin and fur, although the fur was relatively clear and shiny compared with the rats in the model group.

### 3.2. Changes in the Body Weight of Rats and Abdominal Withdrawal Reflex (AWR) Scoring

The body weights of IBS rats after modeling (before treatment) were significantly decreased compared with the body weights of rats in the normal group (*P* < 0.01). After treatment, the body weights of rats in the MM group (*P* < 0.01) and EA group (*P* < 0.05) were significantly higher than the body weights of rats in the model group. However, all IBS rats in different groups had lower body weight than rats in the normal group (*P* < 0.01) (Figure 1(a)). The AWR scores of rats in the model group were significantly elevated under all CRD pressures (20, 40, 60, and 80 mmHg) compared with the normal group (all *P* < 0.01). Compared with the model group, the AWR scores of rats in the MM and PB groups were significantly decreased under 20 mmHg CRD pressure (*P* < 0.05). AWR scores of rats in the MM, EA, and PB groups under 40, 60, and 80 mmHg CRD pressures were significantly decreased (*P* < 0.05 or *P* < 0.01) (Figure 1(b)).

### 3.3. Histological Observation

As shown in Figure 2, the morphology of the colonic mucosa in the normal rats was intact with clear structure, neatly arranged glands, and no inflammatory cell infiltration, congestion, or edema. In the model group, the colonic mucosa of IBS rats still demonstrated regular structure with regularly arranged colonic glands and only small numbers of infiltrated inflammatory cells in the submucosa, and no congestion or edema. Colonic structure of IBS rats in the MM, EA, and PB groups was intact, with relatively neatly arranged glands, few or no inflammatory cell infiltration in the mucosa and submucosa, and no obvious interstitial congestion and edema.

### 3.4. BDNF Protein and mRNA Expression in the Colon

As shown in Figure 3, BDNF protein and mRNA expressions in the colon of IBS rats in the model group were significantly higher than those in the healthy rats in the normal group (*P* < 0.01). Compared with the model group, IBS rats in the MM, EA, and PB groups had significantly lower BDNF protein and mRNA expressions in the colon (*P* < 0.01).

### 3.5. TrkB Protein and mRNA Expression in the Colon

As shown in Figure 4, TrkB protein and mRNA expressions in the colon of IBS rats in the model group were significantly higher than those in the healthy rats in the normal group (*P* < 0.01). Compared with the model group, IBS rats in the MM, EA, and PB groups had significantly lower TrkB protein and mRNA expressions in the colon (*P* < 0.01). In addition, TrkB protein expression in the colon of the MM group was significantly lower than that of the MW group (*P* < 0.01).

### 3.6. BDNF Protein and mRNA Expression in the Dorsal Root Ganglia

As shown in Figure 5, the protein and mRNA expressions of BDNF in the dorsal root ganglia of IBS rats in the model group were significantly higher than those in the healthy rats in the normal group (*P* < 0.01). IBS rats in the MM, EA, and PB groups had significantly lower TrkB protein and mRNA expressions in the dorsal root ganglia than those in the model group (*P* < 0.01).

### 3.7. TrkB Protein and mRNA Expression in the Dorsal Root Ganglia

As shown in Figure 6, the protein and mRNA expressions of TrkB in the dorsal root ganglia of IBS rats in the model group were significantly higher than those in the healthy rats in the normal group (*P* < 0.01). IBS rats in the MM, EA, and PB groups had significantly lower TrkB protein and mRNA expressions in the dorsal root ganglia than those in the model group (*P* < 0.01).

## 4. Discussion

IBS is a chronic functional bowel disease with unclear pathogenesis. Based on the previous research methods, mechanical combined with chemical stimulation were used to simulate the visceral hypersensitivity of IBS in a rat model. Rats in the IBS model group had poor appetite and watery stool, indicating a change in bowel habits. Next, we observed the effect of acupuncture and moxibustion on IBS rats with visceral hypersensitivity and the possible therapeutic mechanism based on BDNF and TrkB. BDNF is one of the neurotrophic factors secreted by spinal microglia and mainly expressed in many brain regions including the cortex and hippocampus. It not only has beneficial effects by promoting the development, survival, and maintenance of neurons in the nervous system but also produces noxious stimuli in the central nervous system and is associated with pain regulation and central sensitization. In addition, BDNF is also abundantly expressed in peripheral gastrointestinal tissues and plays an important role in regulating gastrointestinal motility and visceral sensitivity [23]. Visceral hypersensitivity is an important physiopathological mechanism of IBS [24], and BDNF has been found to promote colon visceral hypersensitivity in animal experiments and clinical studies [25, 26]. The afferent nerves, which innervate intestinal sensation, are mainly distributed in the submucosal plexus and the myenteric plexus. Abnormal BDNF expression in these regions can influence the development of the endplate terminals of the gastrointestinal vagus nerve, thereby affecting the innervation of sensory neurons in the vagus nerve [27]. This allows BDNF to be involved in the modulation of inflammation, occurrence of neuropathic pain, and formation of hypersensitivity in chronic pain [23, 28]. Previous studies have shown that the expression of BDNF protein in the lumbosacral spinal dorsal horn was increased in young mice with visceral hypersensitivity induced by neonatal separation [29], and the mRNA expression of BDNF in the hippocampus of IBS rats with visceral hypersensitivity was significantly higher than that in the normal control rats [30]. After intrathecal injection of BDNF antibody in the dorsal root ganglia of rats with inflammatory pain, the body aches of rats were significantly reduced and the expression level of BDNF in the spinal dorsal horn and hippocampus was also reduced [31], indicating that high BDNF expression in the peripheral nervous system may be an important cause of visceral hypersensitive pain in IBS and other inflammatory pain. The main mechanisms of visceral hypersensitivity are the BDNF-mediated changes in gene expression and channel function in primary sensory neurons and the upregulation of spinal cord BDNF expression which were involved in the development of visceral hypersensitivity induced by prenatal chronic stress [32, 33]. Furthermore, BDNF regulates the integrity of the intestinal epithelial mucosa barrier by affecting the expression of tight junction proteins in the intestinal epithelium, as well as alters the structure of intestinal flora, and is involved in the pathological process of IBS [34, 35].

TrkB, a high-affinity receptor for BDNF, is a tyrosine protein kinase encoded by the thymidine kinase (tdk) proto-oncogene family that can present in the myenteric plexus and submucosal plexus of intestinal tissues. BDNF acts as both an autocrine and a paracrine signal to activate presynaptic TrkB receptors, leading to the activation of tyrosine proteases. The activated tyrosine proteases are involved in the differentiation and development of nerve cells via TrkB-PI3K/AKT, TrkB-MEK/MAPK, and TrkB-PLC/IP3 signaling pathways, and these proteases regulate synaptic excitability in pain conduction and intestinal motility, and they also promote the development of hyperalgesia [36–38]. Binding between BDNF and its receptor TrkB also increases the release of the neurotransmitters serotonin, calcitonin gene-related peptide (CGRP), and P substance (SP) and then causes Ca^2+^ influx on target cell membranes, thereby increasing neuronal discharge activity and excitability in mesenteric afferent nerves and increasing muscle contraction intensity caused by SP and CGRP [39–41]. Studies have found that the expressions of BDNF and nerve fibers were significantly increased in the colon tissues of IBS patients, with damaged ultrastructure of axons in the colon mucosa. BDNF overexpression is also related to the severity and frequency of abdominal pain or discomfort of IBS patients. AWR scores of BDNF-knockout mice under CRD pressure were lower than those of normal mice. Intraperitoneal injection of BDNF in normal mice also induced a dose-dependent increase of postsynaptic TrkB expression and decreased threshold pressure in their dorsal root ganglia [12]. In addition, an IBS rat model induced by repeated water avoidance stress has increased BDNF and TrkB expression in the colon mucosa, submucosa, and myenteric plexus. In that model, BDNF preconditioning enhances the contraction of ring muscle induced by SP, and application of a TrkB antibody inhibited the contraction of colonic muscle. This also attenuates the excitatory effect of SP on the contraction of circular muscle strips, thereby reducing the excessive movement and hypersensitivity of the colon in IBS rats [42]. The above reports suggest that the BDNF-TrkB signaling pathway is closely related to the IBS visceral hypersensitivity, and recent reports also confirmed that blocking BDNF/TrkB signal transduction in IBS model rats attenuated visceral hypersensitivity and synaptic activity [43].

Our results showed that the AWR scores of visceral hypersensitivity in IBS rats were significantly increased. MM and EA treatment reduced AWR scores of IBS rats, suggesting that acupuncture and moxibustion improved the visceral hypersensitivity of IBS rats. In addition, the protein and mRNA expressions of BDNF and TrkB were significantly increased in the submucosal plexus, myenteric plexus, and dorsal root ganglia of IBS rats. MM and EA treatments significantly reduced the AWR scores as well as the protein and mRNA expressions of BNDF and TrkB in the dorsal root ganglia and enteric nervous systems of IBS rats, suggesting that EA and moxibustion may weaken the noxious stimuli and reduce the hypersensitivity of the intestine, thereby achieving their therapeutic effects in IBS.

## Figures and Tables

**Figure 1:** Change of body weight and AWR scores in rats of each group. (a) Weight changes of rats in each group before and after acupuncture and moxibustion treatment. Before treatment, ^*∗*^*P* < 0.01 vs. NC; after treatment, ^*∗*^*P* < 0.01 vs. NC, ^▲^*P* < 0.05 vs. MC, and ^#^*P* < 0.01 vs. MC. (b) AWR scores of rats in each group under different CRD stimulation. ^*∗*^*P* < 0.01 vs. NC, ^▲^*P* < 0.05 vs. MC, and ^#^*P* < 0.01 vs. MC. NC: normal group; MC: model group; MM: model + mild moxibustion group; EA: model + electroacupuncture group; PB: model + pinaverium bromide group.

**Figure 2:** Pathological changes of colon tissue in rats. NC: normal group; MC: model group; MM: model + mild moxibustion group; EA: model + electroacupuncture group; PB: model + pinaverium bromide group (×200).

**Figure 3:** Expression of BDNF protein (×200) and relative expression of BDNF mRNA in rat colon tissue. (a) The expression of BDNF protein in rat colon tissue. (b): The relative expression of BDNF mRNA in rat colon tissue. NC: normal group; MC: model group; MM: model + mild moxibustion group; EA: model + electroacupuncture group; PB: model + pinaverium bromide group. The data were presented as mean ± SD. ^*∗*^*P* < 0.01 vs. NC; ^#^*P* < 0.01 vs. MC.

**Figure 4:** Expression of TrkB protein (×200) and relative expression of TrkB mRNA in the rat colon. (a) Expression of TrkB protein in rat colon tissue. (b) The relative expression of TrkB mRNA in rat colon tissue. NC: normal group; MC: model group; MM: model + mild moxibustion group; EA: model + electroacupuncture group; PB: model + pinaverium bromide group. The data were presented as mean ± SD. ^*∗*^*P* < 0.01 vs. NC; ^#^*P* < 0.01 vs. MC.

**Figure 5:** Expression of BDNF protein (×200) and relative expression of BDNF mRNA in the dorsal root ganglia of rats in each group. (a) Expression of BDNF protein in the dorsal root ganglia of rats. (b) The mRNA expression of BDNF in the dorsal root ganglia of rats. NC: normal group; MC: model group; MM: model + mild moxibustion group; EA: model + electroacupuncture group; PB: model + pinaverium bromide group. The data were presented as mean ± SD. ^*∗*^*P* < 0.01 vs. NC; ^#^*P* < 0.01 vs. MC.

**Figure 6:** Expression of TrkB protein (×200) and relative expression of TrkB mRNA in the dorsal root ganglia of rats in each group. (a) Expression of TrkB protein in the dorsal root ganglia of rats. (b) The mRNA expression of TrkB in the dorsal root ganglia of rats in each group. NC: normal group; MC: model group; MM: model + mild moxibustion group; EA: model + electroacupuncture group; PB: model + pinaverium bromide group. The data were presented as mean ± SD. ^*∗*^*P* < 0.01 vs. NC; ^#^*P* < 0.01 vs. MC.

## Data Availability

The data sets used to support the findings of this study are available from the corresponding author upon reasonable request.

## References

[1] Gupta A. (2013). Peripheral mechanisms in irritable bowel syndrome. *New England Journal of Medicine*.

[2] Wernersson R., Carlsson J. (2015). Posttraumatic stress disorder is correlated to irritable bowel syndrome. *Ugeskrift for Laeger*.

[3] Spiller R., Lam C. (2012). An update on post-infectious irritable bowel syndrome: role of genetics, immune activation, serotonin and altered microbiome. *Journal of neurogastroenterology and motility*.

[4] Cohen-Cory S., Kidane A. H., Shirkey N. J., Marshak S. (2010). Brain-derived neurotrophic factor and the development of structural neuronal connectivity. *Developmental neurobiology*.

[5] Ulmann L., Hatcher J. P., Hughes J. P. (2008). Up-regulation of P2X4 receptors in spinal microglia after peripheral nerve injury mediates BDNF release and neuropathic pain. *Journal of Neuroscience*.

[6] Lever I. J., Bradbury E. J., Cunningham J. R. (2001). Brain-derived neurotrophic factor is released in the dorsal horn by distinctive patterns of afferent fiber stimulation. *The Journal of Neuroscience*.

[7] Steinkamp M., Schulte N., Spaniol U., Pflüger C., Kirsch J., von Boyen G. B. (2012). Apoptosis in enteric glia:Part of the puzzle in Crohn’s disease?. *Medical Science Monitor*.

[8] Lucini C., Maruccio L., De Girolamo P., Castaldo L. (2003). Brain-derived neurotrophic factor in higher vertebrate pancreas: immunolocalization in glucagon cells. *Anatomy and Embryology*.

[9] Wang P., Chen F.-X., Du C. (2015). Increased production of BDNF in colonic epithelial cells induced by fecal supernatants from diarrheic IBS patients. *Scientific Reports*.

[10] Moloney R. D., Dinan T. G., Cryan J. F. (2015). Strain-dependent variations in visceral sensitivity: relationship to stress, anxiety and spinal glutamate transporter expression. *Genes, Brain and Behavior*.

[11] Sikandar S., Minett M. S., Millet Q. (2018). Brain-derived neurotrophic factor derived from sensory neurons plays a critical role in chronic pain. *Brain*.

[12] Yu Y.-B., Zuo X.-L., Zhao Q.-J. (2012). Brain-derived neurotrophic factor contributes to abdominal pain in irritable bowel syndrome. *Gut*.

[13] Wu X. L., Wang Y. L., Sun J. H. (2013). Clinical observation on acupuncture for diarrhea-predominant irritable bowel syndrome patients in syndrome of liver-stagnation and spleen-deficiency and its impact on Th1/Th2. *Zhongguo zhen jiu*.

[14] Anastasi J. K., McMahon D. J., Kim G. H. (2009). Symptom management for irritable bowel syndrome. *Gastroenterology Nursing*.

[15] Manheimer E., Cheng K., Wieland L. S. (2012). Acupuncture for treatment of irritable bowel syndrome. *Cochrane Database of Systematic Reviews*.

[16] Al-Chaer E. D., Kawasaki M., Pasricha P. J. (2000). A new model of chronic visceral hypersensitivity in adult rats induced by colon irritation during postnatal development. *Gastroenterology*.

[17] Wang L. D., Zhao J. M., Huang R. J. (2016). Study on the mechanism underlying the regulation of the NMDA receptor pathway in spinal dorsal horns of visceral hypersensitivity rats by moxibustion. *Evidence-Based Complementary and Alternative Medicine*.

[18] Bao C.-H., Wang C.-Y., Li G.-N. (2019). Effect of mild moxibustion on intestinal microbiota and NLRP6 inflammasome signaling in rats with post-inflammatory irritable bowel syndrome. *World Journal of Gastroenterology*.

[19] Wang X., Wu H., Jin X. (2018). Gut microbiota was modulated by moxibustion stimulation in rats with irritable bowel syndrome. *Chinese Medicine*.

[20] Qi Q., Wu H. G., Jin X. M. (2019). Effect of moxibustion on the expression of GDNF and its receptor GFR*α*3 in the colon and spinal cord of rats with irritable bowel syndrome. *Acupuncture in Medicine*.

[21] Wei W., Wu X., Li Y. (2010). *Experimental Methodology of Pharmacology*.

[22] Li Z.-Y., Huang Y., Yang Y.-T. (2017). Moxibustion eases chronic inflammatory visceral pain through regulating MEK, ERK and CREB in rats. *World Journal of Gastroenterology*.

[23] Coull J. A. M., Beggs S., Boudreau D. (2005). BDNF from microglia causes the shift in neuronal anion gradient underlying neuropathic pain. *Nature*.

[24] Öhman L., Simrén M. (2010). Pathogenesis of IBS: role of inflammation, immunity and neuroimmune interactions. *Nature Reviews Gastroenterology & Hepatology*.

[25] Fu Y., Lin Y. M., Winston J. H., Radhakrishnan R, Huang L. M, Shi X. Z (2018). Role of brain-derived neurotrophic factor in the pathogenesis of distention-associated abdominal pain in bowel obstruction. *Neuro-Gastroenterology and Motility: The Official Journal of the European Gastrointestinal Motility Society*.

[26] Zhang Y., Qin G., Liu D.-R., Wang Y., Yao S.-K. (2019). Increased expression of brain-derived neurotrophic factor is correlated with visceral hypersensitivity in patients with diarrhea-predominant irritable bowel syndrome. *World Journal of Gastroenterology*.

[27] Biddinger J. E., Fox E. A. (2014). Reduced intestinal brain-derived neurotrophic factor increases vagal sensory innervation of the intestine and enhances satiation. *Journal of Neuroscience*.

[28] Liu M., Kay J. C., Shen S., Qiao L.-Y. (2015). Endogenous BDNF augments NMDA receptor phosphorylation in the spinal cord via PLC*γ*, PKC, and PI3K/Akt pathways during colitis. *Journal of Neuroinflammation*.

[29] Wu B., Xu C., Huang H. (2016). Expression profiles of brain-derived neurotrophic factor in the spinal dorsal horn of young rats with visceral hypersensitivity. *Chinese Journal of Contemporary Pediatrics*.

[30] Zhao Y., Su M., Wang F. (2015). Effect of chang’an No.I recipe on 5-hydroxytryptamine signal system and mRNA expression levels of hippocampal brain derived neurotrophic factor in visceral hypersensitivity rats with irritable bowel syndrome. *Chinese Journal of Integrated Traditional and Western Medicine*.

[31] Duric V., McCarson K. E. (2007). Neurokinin-1 (NK-1) receptor and brain-derived neurotrophic factor (BDNF) gene expression is differentially modulated in the rat spinal dorsal horn and hippocampus during inflammatory pain. *Molecular Pain*.

[32] Shi X.-Z., Lin Y.-M., Hegde S. (2018). Novel insights into the mechanisms of abdominal pain in obstructive bowel disorders. *Frontiers in Integrative Neuroscience*.

[33] Winston J. H., Li Q., Sarna S. K. (2014). Chronic prenatal stress epigenetically modifies spinal cord BDNF expression to induce sex-specific visceral hypersensitivity in offspring. *Neuro-Gastroenterology and Motility*.

[34] Yu Y. B., Zhao D. Y., Qi Q. Q. (2017). BDNF modulates intestinal barrier integrity through regulating the expression of tight junction proteins. *Neuro-Gastroenterology and Motility: The Official Journal of the European Gastrointestinal Motility Society*.

[35] Li C., Cai Y.-Y., Yan Z.-X. (2018). Brain-derived neurotrophic factor preserves intestinal mucosal barrier function and alters gut microbiota in mice. *The Kaohsiung Journal of Medical Sciences*.

[36] Lim J. Y., Park S. I., Oh J. H. (2008). Brain‐derived neurotrophic factor stimulates the neural differentiation of human umbilical cord blood‐derived mesenchymal stem cells and survival of differentiated cells through MAPK/ERK and PI3K/Akt‐dependent signaling pathways. *Journal of Neuroscience Research*.

[37] Chen F., Yu Y., Wang P. (2014). Brain-derived neurotrophic factor accelerates gut motility in slow-transit constipation. *Acta Physiologica*.

[38] Lin Y.-T., Ro L.-S., Wang H.-L., Chen J.-C. (2011). Up-regulation of dorsal root ganglia BDNF and trkB receptor in inflammatory pain: an in vivo and in vitrostudy. *Journal of Neuroinflammation*.

[39] Boesmans W., Gomes P., Janssens J., Tack J., Berghe P. V. (2008). Brain-derived neurotrophic factor amplifies neurotransmitter responses and promotes synaptic communication in the enteric nervous system. *Gut*.

[40] Chen F. X., Yu Y. B., Yuan X. M., Zuo X. L, Li Y. Q (2012). Brain-derived neurotrophic factor enhances the contraction of intestinal muscle strips induced by SP and CGRP in mice. *Regulatory Peptides*.

[41] Wang P., Du C., Chen F.-X. (2016). BDNF contributes to IBS-like colonic hypersensitivity via activating the enteroglia-nerve unit. *Scientific Reports*.

[42] Quan X., Luo H., Fan H. (2015). Brain-derived neurotrophic factor contributes to colonic hypermotility in a chronic stress rat model. *Digestive Diseases and Sciences*.

[43] Fan F., Tang Y., Dai H. (2020). Blockade of BDNF signalling attenuates chronic visceral hypersensitivity in an IBS‐like rat model. *European Journal of Pain*.

